The article "Structure-based virtual screening of Trachyspermum ammi metabolites targeting acetylcholinesterase for Alzheimer’s disease treatment" was retracted in 2025. Reasons: unreliable results or conclusions; concerns about the peer review; concerns about the authorship.

# Structure-based virtual screening of *Trachyspermum ammi* metabolites targeting acetylcholinesterase for Alzheimer’s disease treatment

**DOI:** 10.1371/journal.pone.0311401

**Published:** 2024-12-17

**Authors:** Mohammed Sakib Musa, Md. Tahsinul Islam, Wasif Billah, Md. Siam Hossain, Md. Shirajuce Shalakin Rahat, Imren Bayil, Yeasmin Akter Munni, Sumon Ganguli

**Affiliations:** 1 Department of Applied Chemistry and Chemical Engineering, Faculty of Science, University of Chittagong, Chittagong, Bangladesh; 2 Department of Biochemistry and Biotechnology, North South University, Dhaka, Bangladesh; 3 Department of Pharmacy, Faculty of Basic Medicine and Pharmaceutical Science, University of Science and Technology Chittagong, Chittagong, Bangladesh; 4 Department of Pharmacy, Noakhali Science and Technology University, Noakhali, Bangladesh; 5 Department of Pharmacy, University of Rajshahi, Rajshahi, Bangladesh; 6 Department of Bioinformatics and Computational Biology, Gaziantep University, Gaziantep, Turkey; 7 Department of Anatomy, College of Medicine, Dongguk University, Gyeongju, Seoul, Republic of Korea; Cholistan University of Veterinary and Animal Sciences, PAKISTAN

## Abstract

In recent decades, Alzheimer’s disease (AD) has garnered significant attention due to its rapid global prevalence. The cholinergic hypothesis posits that the degradation of acetylcholine by acetylcholinesterase (AChE) contributes to AD development. Despite existing anti-AChE drugs, their adverse side effects necessitate new agents. This study analyzed 150 bioactive phytochemicals from *Trachyspermum ammi* using structure-based drug design and various in-silico tools to identify potent anti-AChE compounds. Compounds were screened for drug-likeness (QEDw ≥50%) and bioavailability (≥55%) and underwent toxicity profiling via the ProTox-II server. Selected compounds were prepared for molecular docking with the human AChE protein as the receptor. Viridifloral, 2-Methyl-3-glucosyloxy-5-isopropyl phenol, Alpha-Curcumene, and Sterol emerged as top candidates with high AChE affinity. These results were validated by molecular dynamics simulations, confirming stable interactions. The hit compounds were further evaluated for drug-likeness using Lipinski’s rule and ADMET properties, confirming favorable pharmacokinetic profiles. DFT optimization analyzed frontier molecular orbitals and electrostatic potential, demonstrating favorable chemical reactivity and stability. This study suggests that these identified compounds could be novel nature-derived AChE inhibitors, potentially contributing to AD treatment. However, further in-vitro and in-vivo studies are necessary to confirm their efficacy in biological systems. Future research will focus on developing these compounds into safe and effective drugs to combat Alzheimer’s disease.

The article "Structure-based virtual screening of Trachyspermum ammi metabolites targeting acetylcholinesterase for Alzheimer’s disease treatment" was retracted in 2025. Reasons: unreliable results or conclusions; concerns about the peer review; concerns about the authorship.

## 1. Introduction

Alzheimer’s disease (AD), the most prevalent dementia-related condition, was first recognized by Alois Alzheimer in 1907 and currently affects approximately 30 million people worldwide, with the number rapidly increasing [1]. AD is characterized by symptoms such as difficulties with perception, reasoning, planning, and thinking. The disease is a complex condition influenced by numerous factors, and despite extensive research, the precise mechanisms underlying its pathogenesis remain unclear due to the intricacies of the human brain, the lack of adequate animal models, and the limitations of current research tools [2]. Several hypotheses have been proposed regarding the development of AD, including those centred on amyloid β (Aβ) accumulation, tau protein tangles, cholinergic neuron damage, oxidative stress, and neuroinflammation. Although extensive research has largely supported the idea that Aβ is a key initiator of the pathogenic cascade in AD, increasing evidence suggests that Aβ is necessary but not sufficient in the later stages of the disease [3].

Efforts to target tau in AD have focused on inhibiting tau aggregation, employing tau-based vaccinations, stabilizing microtubules, and modulating kinases and phosphatases that regulate tau modifications [2]. However, most of these efforts have not succeeded in clinical trials. For instance, the tau aggregation inhibitor TRx0237 did not demonstrate therapeutic benefits in phase III trials [4] and intravenous immunoglobulin (IVIG), the only passive vaccine to reach phase III clinical trials, failed to achieve the primary endpoints in patients with mild-to-moderate AD [5]. Other tau-targeting strategies, such as stabilizing microtubules and modulating kinases and phosphatases, remain in preclinical studies. Tau-targeting therapies present significant challenges due to the incomplete understanding of AD, the lack of robust and sensitive biomarkers for accurate diagnosis and treatment monitoring, and the difficulty of overcoming the blood-brain barrier [2].

Conversely, the strategy of acetylcholinesterase (AChE) inhibition, derived from the cholinergic hypothesis, provides symptomatic relief, albeit with limited benefits. It remains the most widely used and available clinical treatment, offering some hope to AD patients [2]. The cholinergic hypothesis suggests that AD may be caused by the loss of function in cholinergic neurons, leading to impaired cholinergic signalling and neurotransmission in the brain [6]. This hypothesis centres on acetylcholine (ACh), a key neurotransmitter regulated by the enzymes choline acetyltransferase (ChAT) and AChE [7]. AChE’s primary function is to rapidly hydrolyze ACh into acetate and choline, terminating impulse transmission at cholinergic synapses [8]. The enzyme’s active site contains two subsites: the ‘esteratic’ and ‘anionic’ subsites, serving as the catalytic and choline-binding sites, respectively, located in the enzyme’s deep and narrow gorge [9]. AChE has garnered significant attention due to its high catalytic activity (25,000 reactions/second) [10]. Given that defects in cholinergic neurotransmission are linked to AD, cholinesterase inhibitors such as galantamine, donepezil, rivastigmine, and huperzine A have been extensively studied as symptomatic treatments for AD [11, 12].

The article "Structure-based virtual screening of Trachyspermum ammi metabolites targeting acetylcholinesterase for Alzheimer’s disease treatment" was retracted in 2025. Reasons: unreliable results or conclusions; concerns about the peer review; concerns about the authorship.

Although some organophosphate inhibitors have been used as insecticides and chemical warfare agents due to their irreversible inhibition of AChE, resulting in lethal consequences [13], other AChE inhibitor-based drugs have been approved by the FDA, including biperiden, memantine, edrophonium, neostigmine, caproctamine, and tacrine [14, 15]. These drugs are used in treating neurological disorders designed to address cholinergic dysfunction and improve cholinergic efficiency, providing persistent therapeutic effects [16]. However, several of these drugs have been associated with adverse side effects. Tacrine, for instance, was found to have hepatotoxic effects [17], while others have been reported to cause gastrointestinal side effects, such as nausea, diarrhoea, and a rise in cardiac vagal tone that could lead to bradycardia [18, 19]. Rivastigmine and galantamine were also associated with anorexia, headache, diarrhoea, nausea, vomiting, dizziness, abdominal pain, and syncope [20, 21]. Therefore, there is a need for safe and effective AChE inhibitors that can halt the progression of the disease at its initial stage, prevent neurodegeneration, or improve cognitive impairment to reduce the social and financial burden of caring for AD patients and enhance their quality of life [22].

Natural product-derived agents have demonstrated remarkable efficacy as therapeutic agents in neurodegenerative disorders due to their antioxidative, antiapoptotic, anti-amyloidogenic, and modulatory effects on mitochondrial function [23, 24]. Additionally, emerging research suggests that these agents may counteract protein misfolding, affect proteasomal degradation, promote aggregate clearance, and enhance autophagy [25, 26]. For example, the dichloromethane sub-extract (UaD) of *Uvaria alba*, an endemic plant, has shown anti- AChE activity in-vitro [27]. Compounds such as 3-(3,4-dihydroxybenzyl)-3′,4′,6-trihydroxy-2,4-dimethoxychalcone and grandifloracin derived from the plant exhibited strong binding affinity to AChE.

The article "Structure-based virtual screening of Trachyspermum ammi metabolites targeting acetylcholinesterase for Alzheimer’s disease treatment" was retracted in 2025. Reasons: unreliable results or conclusions; concerns about the peer review; concerns about the authorship.

Various plant-based phytoconstituents, including alkaloidal, polyphenolic, and terpenoid compounds, possess excellent therapeutic potential. The Apiaceae family’s *Trachyspermum ammi* L. is a highly valuable medicinal spice with numerous reported pharmacological activities, such as antifungal, antioxidant, antimicrobial, antinociceptive, cytotoxic, hypolipidemic, antihypertensive, antispasmodic, bronchodilating, antilithiasis, diuretic, abortifacient, antitussive, nematicidal, anthelmintic, and antifilarial properties [28]. Additionally, *T*. *ammi* seed extract has demonstrated neuroprotective and learning/memory-enhancing properties in several studies [29, 30]. Consequently, the current study aims to virtually identify potential phytoconstituents as AChE inhibitors from *T*. *ammi* secondary metabolites, which may modulate cognitive and memory function in AD patients by influencing cholinergic and glutamatergic systems, thereby halting the progression of cognitive impairment.

## 2. Methods

A structure-based drug design approach was employed to analyse 150 bioactive phytochemicals of *T*. *ammi*, utilizing various bioinformatics and in-silico biology tools to identify the most effective anti-AChE agents. Advanced molecular docking and dynamics simulation protocols [31–46] were used to explore the interactions and stability of the ligands with target proteins. The stepwise methods of the study are illustrated in **Fig 1.**

**Fig 1:** Stepwise methods of the overall study.

### 2.1. Screening library of phytochemicals from Indian medicinal plants

For this study, 150 phytochemicals from *Trachyspermum ammi* reported in various analytical analyses were compiled into an Excel sheet using data from the IMPPAT database [47]. The newly created screening database included the following extracted information: PubChem ID, SMILES string, drug-likeness (QEDw) score, bioavailability score, molecular weight, and relevant references for each phytoconstituent.

### 2.2. First-phase screening based on drug-likeness and bioavailability score

A crucial factor to consider while choosing compounds in the early phases of drug development is drug-likeness. Nevertheless, assessing drug-likeness in absolute terms does not fully capture the range of compound quality. Worrisomely, commonly used rules may unintentionally encourage unwanted molecular property inflation by allowing rule-compliant compounds to encroach on their bounds. Weighted quantitative estimate of drug-likeness (QEDw) score was used to filter the druggable compounds from the fresh Excel database in the first place. QEDw is a drug-ability score for small molecules proposed by Bickerton et al. [48]. Bioavailability is also an important aspect of druggable small molecules. In this study, we assessed the bioavailability of each compound using swissADME server [49]. In the first phase, the screening criteria were set at ≥50% for QEDw and ≥55% for Bioavailability score.

The article "Structure-based virtual screening of Trachyspermum ammi metabolites targeting acetylcholinesterase for Alzheimer’s disease treatment" was retracted in 2025. Reasons: unreliable results or conclusions; concerns about the peer review; concerns about the authorship.

### 2.3. Toxicity profiling

Compounds screened in the first phase were assessed for toxicity profiling using ProTox-II server [50]. Five toxicological endpoints, carcinogenicity, mutagenicity, cytotoxicity, immunotoxicity, hepatotoxicity, and oral toxicity class were taken into consideration. Only the compounds that showed negative outcomes in all sorts of toxicological endpoints and had an oral toxicity class of 4 or higher were chosen for further analysis.

### 2.4. Ligand collection, retrieving, and preparation

The compounds that met the criteria in first phase screening and toxicity profiling were considered for generating hit compounds. In this aspect, 3D structures of the compounds were downloaded from the IMPPAT database in mol format. Their structures were cross-checked in the PubChem server using CID. Later these mol files were imported into openbabel, and subjected to energy minimization using mmff94 forcefield. Finally, all the files were converted to pdbqt format in the openbabel interface.

### 2.5. Preparation of receptor protein

The human AChE protein (PDB entry: 4EY7) was employed as the receptor and its X-ray crystal structure was retrieved from the Protein Data Bank. It is a homodimer protein containing chains A, and B with a resolution of 2.35 Å. BIOVIA Discovery studio program (version 2021) was used to prepare the protein by removing all hetero atoms, co-crystalized ligands, and water molecules keeping only chain A. Later it was saved in PDB format. This PDB file was subjected to energy minimization utilizing Swiss-Pdb viewer [51] where computations were carried out *in vacuo* with the GROMOS 96 force field.

### 2.6. Molecular docking and validation of docking protocol

In *in silico* drug design, molecular docking is a crucial step for screening hit compounds from thousands for a specific target. In this study, molecular docking was conducted using the AutoDock Vina program for virtual screening. The individual docking of the phytochemical library against the previously energy-minimized target protein was performed with AutoDock Vina, integrated into the PyRx platform [52]. The Lamarckian genetic algorithm (LGA) was employed as the scoring function. Blind docking was carried out for each energy-minimized ligand against the receptor protein. The grid box was maximized to fully encompass the receptor, with dimensions of 58.81 Å × 61.20 Å × 72.82 Å and centered at -2.91, -40.10, and 30.87 along the x, y, and z axes, respectively.

The article "Structure-based virtual screening of Trachyspermum ammi metabolites targeting acetylcholinesterase for Alzheimer’s disease treatment" was retracted in 2025. Reasons: unreliable results or conclusions; concerns about the peer review; concerns about the authorship.

After successful docking, the ligand binding poses were obtained, and those with the lowest root mean square deviation (RMSD) values were selected for visualization using the Discovery Studio Visualizer program. This visualization allowed for the evaluation of hydrogen bonds, hydrophobic interactions, and pi-interactions. To ensure the accuracy and reliability of the docking process, we implemented a systematic validation approach that included both redocking and alignment techniques. Specifically, for validating the AChE (PDB ID: 4EY7) docking process, the co-crystal ligand (donepezil) was separated and re-docked using the same blind docking parameters. The RMSD value was calculated in PyMOL by aligning the lowest energy docked conformer with the co-crystal ligand. An RMSD value of ≤2 Å (0.2 nm) generally indicates the reliability of a docking method [53]. The calculated RMSD value was 0.077 Å (**S1 Fig**), indicating excellent alignment between the co-crystal and re-docked structures, as the RMSD value is well within the favorable range (≤2 Å). Thus, it can be inferred that using the same docking methodology is likely to produce accurate and reproducible conformers for screening the compound library derived from *T*. *ammi*.

### 2.7. Molecular dynamics simulation analyses

Molecular dynamics (MD) simulations were conducted to assess the accuracy of the molecular docking analyses that were performed. MD simulation is widely recognized as a crucial method for assessing the stability of protein-ligand complexes. It offers valuable insights into the fluctuations and conformational changes that occur, ultimately leading to the identification of the stable conformation [54]. Thus, in the present study, MD simulations of the targeted receptor protein AChE with selected ligand complexes have been conducted to establish the binding accuracy of viridifloral, curcumene, sterol, and control galantamine to the targeted protein. The calculations were carried out for a duration of 200 nanoseconds (ns) in a periodic water box using the Gromacs version 2020 software package and the CHARMM36 force field [55, 56]. With the help of the CHARMM-GUI web-based graphical interface, the simulation system was set up, and the force fields for both the ligands and the protein were created [57]. The complexes were placed inside a rectangular container with a buffer spacing of 10 units in each of the cardinal directions. The box was dissolved in a solution of water molecules containing TIP3P [58]. To ensure system neutrality, salt and chloride ions were introduced into the system, followed by energy minimization using the steepest descent approach. The equilibration procedure was conducted on all complete systems at a temperature of 310 K for a total of 5,000 steps, which is equivalent to 10 picoseconds (PS). The systems were equilibrated using an isothermal-isochoric ensemble NVT, which maintains a constant number of particles, volume, and temperature, and an isothermal-isochoric ensemble NPT, which maintains a constant number of particles, pressure, and temperature. The Lincs method was utilized to limit the presence of hydrogen, resulting in a time step of 2 fs. We performed a thorough evaluation of all Vander Waals (vdw) forces using a switching mechanism that ranged from 12 to 14 Å, with a cut off value of 14. The particle mesh Ewald (PME) approach with a maximum grid spacing of 1.2 has been used to determine the long-term electrostatic interactions. Instead of employing a multiple-time-stepping strategy, PME processes have been executed at each individual step. The temperature remained unchanged at 310 K. The barostat was configured to control variations in system size to a specific level of 1 bar [59, 60]. The integration time step was 2 femtoseconds. After the 200 ns MD simulation was finished, the simulation results were first recentered. Afterwards, the trajectory data were examined using the integrated tools in Gromacs and VMD to study the dynamic conformational changes and interactions within the complexes during the duration [61]. Examined simulated trajectories to compute various metrics such as RMSD, root mean square fluctuation (RMSF), radius of gyration (Rg) growth, number of H-bonds, principal component analysis (PCA), and dynamics cross-correlation matrices (DCCM).

The article "Structure-based virtual screening of Trachyspermum ammi metabolites targeting acetylcholinesterase for Alzheimer’s disease treatment" was retracted in 2025. Reasons: unreliable results or conclusions; concerns about the peer review; concerns about the authorship.

### 2.8. Lipinski’s rule of five and ADMET determination

For the hit compounds along with control ligand, Lipinski’s rule and ADMET properties were assessed to predict their drug-ability. The ADME pharmacokinetic characteristics which are essential for a compound to be a drug, are absent from half of the drug candidates, which lead to their failure in the development process [62]. The pkCSM web server was used to evaluate each of the compounds’ ADMET profile [63]. Selected pharmacokinetic properties i.e., human intestinal absorption, inhibition of cytochrome P450, Blood–Brain Barrier (BBB) penetration, etc. were considered for the evaluation. Using Lipinski’s rule of five, substances that are similar to drugs and those that are not were distinguished. SwissADME server was used to estimate crucial pharmacokinetic parameters such as molecular weight, hydrogen bond donor, hydrogen bond acceptor, and consensus log Po/w. Lipinski’s Rule was also predicted using same web server [49].

### 2.9. DFT optimization

Gaussian 09W Revision (D.01)17 was employed for geometry optimization and further calculations of the hit compounds. In the gas phase, 6-31g (d, p) basis set combined with B3LYP correlation function, and density functional theory (DFT) utilized to study their Frontier molecular orbitals and Molecular electrostatic potential (MEP) [64–67]. The optimized structures are demonstrated in **Fig 2**. Frontier molecular orbitals; ‘Highest Occupied Molecular Orbital’ (HOMO) and ‘Lowest Unoccupied Molecular Orbital’ (LUMO) were determined keeping similar level of theory. Afterward, the HOMO-LUMO energy gap (ΔE), chemical softness (S), chemical hardness (η), chemical potential (μ), and electrophilicity (ω) were determined using the following equations [68–70].


$$\mathrm{Gap}\;(\Delta \text{E})=[\text{L}-\text{H}];\eta =\frac{\Delta \text{E}}{2};S=\frac{1}{\eta }$$

$$\mu =\frac{\left[\text{L}+\text{H}\right]}{2};\chi =-\frac{\left[\text{L}+\text{H}\right]}{2};\omega =\frac{\mu 2}{2\eta }$$

**Fig 2:** DFT optimized structures of the hit compounds.

## 3. Results and discussion

### 3.1. *In silico* chemical profiling and compound library

Initially, a phytochemical library consisting of 150 bioactive compounds derived from *T*. *ammi* was compiled from the IMPPAT database for this study. In the preliminary screening phase, compounds that exhibited poor drug-likeness and bioavailability properties were excluded. From the initial 150 compounds, 102 were selected for further evaluation based on their favorable drug-likeness and bioavailability profiles. The subsequent toxicity assessment revealed that 67 out of the 102 compounds met safety criteria across various toxicological endpoints, including carcinogenicity, mutagenicity, cytotoxicity, immunotoxicity, and hepatotoxicity. Furthermore, these 67 compounds were classified within oral toxicity class 4 or higher, indicating their safety for oral administration. The screening results highlight the importance of choosing compounds with good drug-likeness, bioavailability, and strong safety profiles. While initial screenings identify promising candidates, rigorous toxicity testing is crucial to ensure their suitability for further development. The high toxicity rates among the screened compounds emphasize the need for careful evaluation to select safe and effective candidates for subsequent studies.

### 3.2. Molecular docking and non-bonding interaction analysis

Molecular docking is a crucial technique for predicting the bioactive potential of chemical compounds against target receptors linked to disease states. In this study, 67 phytoconstituents from *T*. *ammi* were analysed using molecular docking, with the results summarized in **S2 Fig**. The optimal docking poses were evaluated based on the lowest binding energy and RMSD values. Curcumene, 2-Methyl-3-glucosyloxy-5-isopropyl phenol, sterol, and viridifloral were selected as the top four hit compounds for their strong binding affinity to the AChE enzyme, as detailed in **Table 1**. Galantamine, a well-established AChE inhibitor used in AD treatment, served as a control to compare the docking results and non-bonding interactions.

The article "Structure-based virtual screening of Trachyspermum ammi metabolites targeting acetylcholinesterase for Alzheimer’s disease treatment" was retracted in 2025. Reasons: unreliable results or conclusions; concerns about the peer review; concerns about the authorship.

**Table 1:** Molecular docking and non-bonding interaction analysis of the top four hit compounds along with reference drug galantamine.

PubChem ID	Ligands	Binding Affinity	Residue in contact	Interaction Type	Bond Distance (Å)
11996452	Viridifloral (VIR)	-10.2	TRP86	PS	2.66537
			TRP86	PA	5.13515
			TRP86	PA	5.20057
			TRP86	PA	4.36722
			TYR124	PA	4.93519
			PHE297	PA	4.54135
			TYR337	PA	5.07537
			TYR337	PA	4.40152
			TYR337	PA	3.62949
			PHE338	PA	3.56295
			PHE338	PA	4.83069
			TYR341	PA	4.48747
			TYR341	PA	4.97489
			HIS447	PA	5.42243
			HIS447	PA	5.19013
129829285	2-Methyl-3-glucosyloxy-5-isopropyl phenol (PHE)	-10	PHE295	H	2.46179
			ARG296	H	2.53734
			SER293, VAL294	APS	4.49675
			LEU289	A	4.83185
			TRP286	PA	4.74972
			TYR341	PA	4.67223
92139	Alpha-Curcumene (CUR)	-9.9	TRP86	PPs	3.90465
			TRP86	PPs	4.21235
			TRP86	PA	4.13694
			TRP86	PA	4.24098
			TYR124	PA	4.9729
			PHE297	PA	5.45062
			PHE297	PA	4.8662
			TYR337	PA	4.83638
			PHE338	PA	5.19556
			PHE338	PA	4.86424
			PHE338	PA	4.84832
			TYR341	PA	4.07474
			TYR341	PA	4.68623
1107	Sterol (STE)	-9.8	TYR124	H	2.73098
			TRP286	PA	4.74031
			TRP286	PA	4.94473
			TRP286	PA	3.79014
			PHE338	PA	4.63987
			TYR341	PA	4.40357
			TYR341	PA	3.82545
			TYR341	PA	5.11418
9651	Galantamine (GAL) Control	-8.9	TYR124	H	2.48923
			TYR124	CH	2.48563
			TYR124	PA	4.90632
			TYR337	PA	5.36371
			PHE338	PA	5.03457
			TYR341	PA	4.99521

H = Conventional hydrogen bond, CH = Carbon Hydrogen Bond, A = Alkyl, PA = Pi-Alkyl, PS = Pi-sigma, PPs = Pi-Pi stacked, APS = Amide-Pi stacked

The docking analysis revealed binding affinities for the screened compounds ranging from -6.3 kcal/mol to -10.2 kcal/mol. Among these, 3-octanol exhibited the lowest affinity, while viridifloral demonstrated the highest affinity. For comparison, galantamine showed a docking score of -8.9 kcal/mol. Further visualization of the docked complexes using Discovery Studio provided insights into ligand-receptor interactions. Analysis of the amino acid residues within 5 Å of the binding site, including Tyr72, Asp74, Tyr124, Trp286, Ser293, Val294, Phe295, Arg296, Phe297, Tyr337, Phe338, and Tyr341, revealed the nature of non-bonding interactions and bond distances (**Fig 3**). The results suggest that the identified hit compounds from T. *ammi* have significant potential as effective AChE inhibitors, potentially paving the way for new therapeutic developments in AD.

The article "Structure-based virtual screening of Trachyspermum ammi metabolites targeting acetylcholinesterase for Alzheimer’s disease treatment" was retracted in 2025. Reasons: unreliable results or conclusions; concerns about the peer review; concerns about the authorship.

**Fig 3:** Docked conformer of Viridiflorol and Alpha-Curcumene interacting in the same binding pocket of receptor protein acetylcholinesterase: (A) Zoomed pose, (B) 3D depiction of non-bonding interaction with the key amino acid residues, (C) Hydrogen bond surface area.

### 3.3. Molecular dynamics simulation analyses

Based on the docking scores, Curcumene, Sterol, Viridifloral, and the control drug Galantamine were chosen for MD simulations to evaluate the stability of their interactions with the AChE enzyme. The MD simulations assessed the stability and dynamics of the ligand-enzyme complexes over time, offering insights into binding stability, conformational changes, and interaction patterns. This analysis helped to confirm the docking results and predict the potential effectiveness of these inhibitors.

#### 3.3.1. Root mean square deviation analysis

RMSD refers to the occurrence of deviations that were noticed during the evolution of the simulation. Furthermore, the RMSD defines the stability of the structural as the smaller the RMSD, the greater the stability [71]. The RMSD calculations were performed on the ligands and complexes throughout a 200 ns MD simulation of each protein-ligand complex. This analysis provided valuable information about the conformational changes that occur during protein-ligand interactions, as depicted in **Fig 4**. Derived from a 200 ns MD simulation, the RMSD of the ligand and complex RMSD values for curcumene, sterol, viridifloral and control galantamine are displayed.

**Fig 4:** (A) RMSD analysis of acetylcholinesterase complexes over a 200 ns MD simulation. The RMSD values are shown for curcumene (black), galantamine (red), sterol (green), and viridifloral (blue). (B) RMSD values of ligands within the selected complexes. (C) RMSF values for the four compounds complexed with acetylcholinesterase during the 200 ns MD simulation. (D) Rg graph for the complexes of curcumene, galantamine, sterol, and viridifloral during the 200 ns MD simulation, shown in black, red, green, and blue respectively.

The stability of each protein-ligand combination was evaluated by calculating the RMSD values of the four complexes across a 200 ns MD trajectory, as depicted in **Fig 4A**. The average absolute RMSD values for the complexes are 1.776 Å, 1.562 Å, 1.339 Å, and 1.471 Å, respectively. The RMSD values of all four complexes exhibit a substantial increase from the initial position of the simulation to the first 10 ns. This increase is particularly strong for galantamine and sterol complexes. Following this period, the RMSD values steadily rose until reaching 20 ns, at which point each complex exhibited minor variations of up to 65 ns. Starting from 65 ns to the end of the simulation, the behaviour of curcumene and galantamine complexes exhibited notable differences when compared to the complexes of sterol and viridifloral. Specifically, the galantamine complex showed a notable increase in RMSD value at 68 ns and 88 ns, reaching its peak during these times. The curcumene complex also exhibited significant changes throughout the simulation, with the highest RMSD value observed around 125 ns. Conversely, sterol and viridifloral complexes exhibit exceptional stability, maintaining a consistent RMSD value until the final 40 ns of the simulation. The simulation results demonstrate that sterol and viridifloral complexes exhibit greater stability and experience fewer conformational changes compared to other complexes (**Fig 4A**).

The article "Structure-based virtual screening of Trachyspermum ammi metabolites targeting acetylcholinesterase for Alzheimer’s disease treatment" was retracted in 2025. Reasons: unreliable results or conclusions; concerns about the peer review; concerns about the authorship.

In addition, upon comparing the ligands based on the RMSD data, it is evident that the curcumene ligand exhibits a significantly higher average RMSD value compared to the galantamine, sterol, and viridifloral ligands (**Fig 4B**). The curcumene ligand has an average RMSD value of 1.378 Å. The protein AChE, bound to the curcumene ligand, did not demonstrate a stable RMSD value for the whole simulation period. Instead, it displayed significant fluctuations during the simulation. At the beginning of the simulation, there was a noticeable increase in the RMSD value for the first 5 ns. It then briefly decreased, but between 10 ns and 20 ns, there was a significant increase in the RMSD value, reaching up to 2 Å. After this increase, although it shows minimal fluctuations until about 60 ns, it shows very large fluctuations in the last 40 ns of the simulation and reaches the highest RMSD value especially at 70 ns and 90 ns. Afterwards, the RMSD value continued to fluctuate and did not reach equilibrium throughout the remainder of the simulation. These findings indicate that the curcumene ligand, when bound to the AChE protein, exhibits a wide range of binding orientations. Additionally, the ligand undergoes positional changes and intermittently exits the binding pocket during the MD simulations. The docking position was considered unacceptable for a candidate with a complex structure. However, the mean RMSD values for galantamine, sterol, and viridifluoral ligands are 0.382 Å, 0.138 Å, and 0.610 Å, respectively. The sterol ligand demonstrates exceptional stability, evidenced by its minimal RMSD value and consistent conformational orientation throughout the simulation. In contrast, when the galantamine ligand is bound, it exhibits a lower RMSD value compared to the viridifloral ligand but undergoes significant fluctuations during the simulation, particularly after the first 15 ns and around 110 ns. Ultimately, it exits the binding site, with pronounced fluctuations occurring during the final 20 ns of the simulation (**Fig 4B**). According to these findings, during the simulation, the binding direction of galantamine ligand changed compared to sterol and viridifloral ligands, and the intermolecular connections changed during the simulation. Furthermore, when the trajectories were analysed with the VMD programme, the results showed that the sterol and viridifluoral ligands do not jump out of the protein domain and are located within the binding site.

The article "Structure-based virtual screening of Trachyspermum ammi metabolites targeting acetylcholinesterase for Alzheimer’s disease treatment" was retracted in 2025. Reasons: unreliable results or conclusions; concerns about the peer review; concerns about the authorship.

#### 3.3.2. Root mean square fluctuation analysis

The RMSF parameter enables the evaluation of the significance of protein residues in the formation of a stable conformation for the protein-ligand complex, providing valuable insights on its stability. A substantial RMSF value indicates higher flexibility, whereas a lower RMSF value suggests more excellent stability. Higher residues or groups in the RMSF plot indicate increased flexibility, thereby offering a higher likelihood of interactions with ligand molecules. Conversely, lower fluctuations in RMSF often signify reduced flexibility, resulting in diminished interaction potential [72]. The RMSF data for the Proteins has been shown in **Fig 4C** to demonstrate the average fluctuation of all amino acid residues over a 200 ns MD trajectory.

The RMSF plot generates a visual depiction defined by prominent peaks, with each peak corresponding to a relatively elevated RMSF value (**Fig 4C**). Based on the RMSF plot, the galantamine compound has the greatest RMSF value and has a significantly greater number of meaningful peaks compared to the other compounds. The peaks were situated among the amino acid ranges of 76–83, 228–250, 265–267, 300–310, 385–389, 433–437, 492–495, and 538–542. Furthermore, these amino acids are part of the binding pocket and have an important influence on the ligand binding process. The larger peak values observed in the galantamine complex suggest that the binding between the ligand and protein is less stable compared to other complexes. The curcumune, sterol, and viridifloral complexes exhibit substantial variations, with prominent peaks observed within the amino acid range of 76–83, 257–258, 322–323, 385–389, 493–494, and 538–542. Furthermore, the RMSF graph of the ligand-protein complex in **Fig 4C** clearly demonstrates a significant increase in the RMSF value at the N-terminal residues corresponding to the tails or ends of the protein structure. The GLU4 (N-terminal) residue exhibited significantly larger fluctuations compared to other residues, particularly showing the highest RMSF value in the galantamine complex. This is probably due to its position at the end of the protein sequence, which gives it more flexibility compared to other amino acid residues. Furthermore, the RMSF values at the C terminal exhibit significant variations among the various complexes. The larger RMSF values seen at the C-terminal ends in the curcumene and galantamine complexes, compared to the other two complexes, can be attributed to the fact that ligand binding weakens the interaction in these complexes, leading to a rise in the RMSF value.

The article "Structure-based virtual screening of Trachyspermum ammi metabolites targeting acetylcholinesterase for Alzheimer’s disease treatment" was retracted in 2025. Reasons: unreliable results or conclusions; concerns about the peer review; concerns about the authorship.

#### 3.3.3. Radius of gyration analysis

To evaluate the changes in structural compression, the diagram of the Rg of each structure was monitored throughout the simulation. The compactness of the system was assessed by calculating the Rg, with higher Rg values indicating lower compactness (more unfolded) with increased conformational entropy and lower Rg values indicating higher compactness with greater structural stability (more folded) [73].

The simulated Rg values for the four complexes are 2.098 Å, 1.978 Å, 1.571 Å, and 1.675 Å, respectively, as shown in **Fig 4D**. Overall, the changes in Rg values for the curcumene and galantamine complexes show significant differences compared to those of the sterol and viridifloral complexes. The curcumene and galantamine complexes exhibited the highest Rg values, with the curcumene complex peaking at 73 ns and 95 ns, and the galantamine complex reaching its highest Rg value at 174 ns. This suggests a relatively weak binding affinity between the ligands and the active site in both cases. In contrast, the sterol and viridifloral complexes displayed minimal variations during the simulation, indicated by their lower Rg values, suggesting these complexes were stable and maintained a compact structure.

#### 3.3.4. Hydrogen bond analysis

During the simulation, we analysed the stability of hydrogen bonds (Hbonds) in protein-ligand complexes, in addition to conducting RMSD, RMSF, and RG analyses. The quantity of hydrogen bonds formed between the ligand molecule and the proteins was computed and illustrated in a graph, as presented in **Fig 5A**. Stabilizing protein-ligand complexes is dependent on the intermolecular H-bonding between the protein and ligand. Throughout the 200 ns simulation period, the stability of the H-bond network formed between proteins and ligands has been calculated. It was anticipated that the quantity of formed H-bonds would depend on the duration of the simulation, indicating the stability of the system during the simulation. In this study, the criteria for hydrogen bonding were established based on the acceptor-donor distance being less than 0.30 nm and the angle being greater than 120 degrees. It is worth noting that a distance of 0.30 nm is commonly used in the scientific literature to define hydrogen bonds [74].

The article "Structure-based virtual screening of Trachyspermum ammi metabolites targeting acetylcholinesterase for Alzheimer’s disease treatment" was retracted in 2025. Reasons: unreliable results or conclusions; concerns about the peer review; concerns about the authorship.

**Fig 5:** (A) Number of hydrogen bonds contributing to the stability of the Galantamine, Sterol, and Viridifloral complexes over 100 ns. (B) Projection of Cα atoms in the essential subspace along the first two eigenvectors for the ligands Curcumene (black), Galantamine (red), Sterol (green), and Viridifloral (blue).

Utilizing the VMD H-bonding analysis tool, all conceivable hydrogen bonding interactions between the two specified areas—such as the protein and the ligand—have been explored over time. The analysis computes the total number of H-bonds and their occupancy throughout the duration. These values are available from the ’Percentage occupancy of the H-bond’ output of the H-bond analysis tool. The ’Percentage occupancy of the H-bond’ output provides these critical metrics [74].

During the molecular dynamics (MD) simulations, hydrogen bonds in the docking structures were maintained in both the sterol and galantamine complexes, with the formation of new hydrogen bonds also observed. **Table 2** details the individual occupancy of detected H-bonds per ligand for, Galantamine, Sterol, and Viridifloral. Hydrogen bonds play a crucial role in identifying non-bonding interactions between proteins and ligands by indicating these interaction.

**Table 2:** H–bonds formed by the ligand molecule with the targeted proteins.

Complexes	Donor-Acceptor	Occupancy
Curcumune	TYR382-Side-OH ASP404-Side-OD2	99%
	ARG152-Side-NE ASP175-Side-OD2	98.50%
Galantamine	TYR382-Side-OH ASP404-Side-OD2	136.56%
	TRP117-Main-N VAL147-Main-O	116.88%
	LEU115-Main-N VAL145-Main-O	113.49%
Sterol	ASN100-Main-N SER148-Main-O	96.60%
	VAL326-Main-N ARG424-Main-O	87.91%
Viridifloral	LEU536-Main-N PHE531-Main-O	117.79%
	ARG246-Side-NH2 VAL288-Main-O	118.69%

The stability of the curcumene complex was maintained through interactions with TYR 382 and ARG 152 residues, with hydrogen bonding between curcumene and TYR 382 showing a maximum occupancy of 99%. The occupancy was 98.50% with curcumene acting as a donor to ARG 152. For the galantamine complex, stability during molecular dynamics simulations was maintained by interactions with TYR 382, TRP 117, and LEU 115 residues. The complex exhibited hydrogen bonds with the highest occupancy at 136.56%, where galantamine formed a bond with TYR 382. Additionally, with 116.88% occupancy, galantamine acted as an acceptor to TRP 117, and LEU 115 contributed with a 113.49% occupancy. Galantamine maintained the hydrogen bond identified in docking simulations, with the formation of additional hydrogen bonds also observed. Sterol formed more hydrogen bonds compared to galantamine, with the highest occupancy at 96.60%, where sterol and ASN 100 formed hydrogen bonds. Another occupancy was at 87.91%, where sterol acted as a donor to VAL 326. For the viridifloral complex, the highest hydrogen bond occupancy was observed at 118.69%, with viridifloral acting as an acceptor to ARG 246, and 117.79% with LEU 536. The hydrogen bonds formed persisted throughout the 200 ns simulation, with particularly high occupancy observed after 100 ns. The viridifloral complex exhibited the highest number and occupancy of hydrogen bonds, suggesting it is more stable than the curcumene, galantamine, and sterol complexes. The stability of each system is determined by the total number and occupancy of these hydrogen bonds, which directly influence the stability of the protein-ligand complex during MD simulations.

The article "Structure-based virtual screening of Trachyspermum ammi metabolites targeting acetylcholinesterase for Alzheimer’s disease treatment" was retracted in 2025. Reasons: unreliable results or conclusions; concerns about the peer review; concerns about the authorship.

#### 3.3.5. Principal component analysis and energy landscape analysis

PCA is a valuable methodology for extracting significant insights from MD trajectories through the segregation of global slow motions from local fast motions [75]. The utilization of principal component analysis (PCA) has facilitated the detection of conformational changes in protein-ligand structures as well as the identification and comprehension of significant coherent motions in diverse regions. Furthermore, this technique can be employed to investigate the impact of diverse parameters on collective movement and simplify the intricacy of motion, which is associated with the steadiness of the system and the functions of complex systems. It is useful to predict important movements in orbit [76]. To gain a deeper understanding of how protein dynamics can affect the binding of ligands, we employed principal component analysis (PCA) to identify the key molecular movements in each of the four simulations. The eigenvectors, referred to as the basic components, were initially computed for the backbone atoms of each trajectory. Afterwards, each trajectory was aligned with the apo eigenvectors for comparative analysis [77]. The spatial covariance matrix was computed for the eigenvectors and their atomic coordinates. An orthogonal coordinate transformation was employed to generate a diagonal matrix of eigenvalues. From these eigenvectors and eigenvalues, the principal components were extracted (**Fig 5B**). Utilizing these principal components, the dominant motions during the simulation were plotted. **Fig 6** illustrates the overall movement of all the protein-ligand complexes (PLCs) using the first two principal components (PCs) and their two-dimensional projections on PC1 and PC2.

The article "Structure-based virtual screening of Trachyspermum ammi metabolites targeting acetylcholinesterase for Alzheimer’s disease treatment" was retracted in 2025. Reasons: unreliable results or conclusions; concerns about the peer review; concerns about the authorship.

**Fig 6:** Free energy landscapes of four crystal structures during 200 ns MD simulation. 2D and 3D graphs projected on the first two principal components (PC1 + PC2). Blue spots indicate the energy minima. Gibbs free energy landscape obtained during 200 ns dynamics of (A) Curcumene (B) Galantamine, (C) Sterol and (D) Viridifloral.

The two principal components (PC1 and PC2) of the sterol and viridifloral complexes, compared with the curcumene and galantamine complexes, showed that the viridifloral complex occupies a smaller region in the conformational space. In contrast, the curcumene complex spans the largest conformational space, indicating increased protein flexibility upon ligand binding. However, after binding with viridifloral, the target protein stabilized and occupied a smaller conformational space, indicating reduced protein flexibility (**Fig 6**).

To identify the low-energy basins (minima) explored during the 200 ns simulation, a free energy landscape (FEL) analysis was conducted. The FEL was graphed in both 2D and 3D using PC1 and PC2. For the free energy landscape, the color gradient represents the frequency or probability of the protein being in a particular conformation, with red areas indicating low probability (high energy) states and blue areas indicating high probability (low energy) states. The simulation reveals that protein-ligand complexes with shallow and narrow energy basins are less stable in terms of structural integrity. As Gibbs free energy decreases, the stability of the conformation and the system increases. The results show that sterol and viridifloral complexes have more low-energy conformations than curcumene and galantamine. These conformations are depicted in the dark blue areas of **Fig 6C and 6D**, indicating thermodynamically favorable positions. The valleys for both sterol and viridifloral complexes were wider, with most energy minima having tapered ends, indicating more stable shapes. In contrast, the energy basins of the curcumene and galantamine complexes were less prominent and narrower (**Fig 6A and 6B**). These findings demonstrate that sterol and viridifloral complexes exhibit remarkable stability.

#### 3.3.6. Dynamic cross‑ correlation matrix analysis

The interrelated structural movements of the complexes were further examined using the DCCM technique, which investigates the motion of the individual components within the system. **Fig 7** displays a red zone indicating a highly positive region with a strong correlation in the movement of the residues in the same direction. Conversely, the blue zone indicates a negative region with anti-correlated motion of the residues. The depth of the colour represents the degree of movement of the atoms [78].

The article "Structure-based virtual screening of Trachyspermum ammi metabolites targeting acetylcholinesterase for Alzheimer’s disease treatment" was retracted in 2025. Reasons: unreliable results or conclusions; concerns about the peer review; concerns about the authorship.

**Fig 7:** DCCM of the Cα atoms plots for 200 ns of (A) curcumene, (B) galantamine, (C) sterol, and (D) viridifloral. Positive (red) and negative (blue) correlations are determined by analyzing the relative movements of the residues. A positive correlation indicates that the residues move in the same direction, while a negative correlation indicates that they move in opposite directions. Uncorrelated movement, represented by the color white, refers to residual movement that does not have an impact on the movement of others.

Upon comparing the DCCM diagrams of the four systems, it becomes evident that the correlation behaviour of the curcumene and galantamine complexes differs dramatically from that of the sterol and viridifloral complexes. Both systems have a notable rise in negative correlation movements, as indicated in the black boxes, while the positive correlation declines. This rise signifies substantial alterations in protein-related movements subsequent to the binding of a ligand. Upon analysing the DCCM diagrams of the curcumene and galantamine systems, it is evident that there is no noteworthy disparity in the correlation motions. The existence of negatively linked movements in these systems implies that the protein’s structural condition is extremely unstable, particularly following interaction with a ligand. According to the research, the viridifloral complex demonstrates the highest level of correlated motion compared to the other complexes. Specifically, the viridifluoral complex exhibited a higher degree of both correlated and anti-correlated motions, suggesting the presence of more and stronger cross-correlation motions. This ultimately results in a stronger connection and improved stability of the complex.

#### 3.3.7. Binding free energy calculation using MM-PBSA

In MD simulations, free energy calculations are crucial for determining the binding stability of ligand-protein complexes. The MM-PBSA approach was employed in this study to compute the free interaction energy between ligands and the specific receptor protein AChE. This approach considers both bonded and non-bonded interactions, including van der Waals and electrostatic forces. Binding free energy (ΔG) estimation was done using the MMPBSA.py script from the AMBER package [79], based on the following equation:

$$\Delta G_{bind}=G_{complex}-\left(G_{receptor}+G_{ligand}\right)$$

Where, *G*_*bind*_ is the free energy of the complex; *G*_*receptor*_ is the free energy of the receptor; *G*_*ligand*_ is the free energy of the ligand [80].

The article "Structure-based virtual screening of Trachyspermum ammi metabolites targeting acetylcholinesterase for Alzheimer’s disease treatment" was retracted in 2025. Reasons: unreliable results or conclusions; concerns about the peer review; concerns about the authorship.

An extensive analysis was conducted using the molecular mechanics Poisson-Boltzmann surface area (MM-PBSA) method to calculate the binding free energy and examine the molecular interactions and stability of the ligand-protein complexes curcumene, galantamine, sterol, and viridifloral with the target receptor protein AChE.

This analysis provides valuable insights into the complex mechanisms underlying its binding and stability [73]. The greater the negative values, the more favorable the binding free energy between proteins and ligands [71]. **Table 3** and **Fig 8** present the free binding energies of the ligands, which are −17.48 ± 3.30 kJ/mol for curcumene, −17.55 ± 2.76 kJ/mol for galantamine, − 21.85 ± 2.08 kJ/mol for sterol, and -16.91 ± 3.35 kJ/mol for viridifloral. The van der Waals energy (EvdW) plays a significant role in the binding of galantamine, sterol, and viridifluoral ligands to the protein. Conversely, the polar energy has an adverse effect with a positive value. **Table 3** indicates that the electrostatic energy and van der Waals interactions have a substantial role in determining the free binding energies of the complexes. This indicates that the sterol complex has the strongest binding free energy compared to the other complexes.

**Fig 8:** Binding free energy plot of (A) curcumene, (B) galantamine, (C) sterol, and (D) viridifloral.

**Table 3:** Binding free energy results of (A) curcumene, (B) galantamine, (C) sterol and (D) viridifloral.

Compounds	ΔEVDW (kJ/mol)	ΔEEEL (kJ/mol)	ΔGPB (kJ/mol)	ΔGNP (kJ/mol)	ΔGDISP (kJ/mol)	ΔG Binding (kJ/mol)
**Curcumene**	-24.77	-0.95	10.99	-2.76	0.00	-17.48 ± 3.30
**Galantamine**	-33.55	-188.13	207.68	-3.56	0.00	-17.55 ± 2.76
**Sterol**	-35.82	-7.35	23.66	-3.37	0.00	-21.85 ± 2.08
**Viridifloral**	-26.89	-6.44	19.48	-3.08	0.00	-16.91 ± 3.35

### 3.4. Lipinki’s rule analysis

The "rule-of-five," established by Lipinski and colleagues, is a widely recognized guideline used to predict the oral bioavailability of pharmaceutical compounds. This rule, developed from an analysis of 2,245 drugs that had advanced to Phase II trials, suggests that compounds may face absorption challenges if they meet two or more of the following criteria: (1) Molecular weight (MW) greater than 500 Da, (2) More than 10 hydrogen-bond acceptors (HBA), (3) More than 5 hydrogen-bond donors (HBD), (4) Calculated logP greater than 5.0 (using ClogP) or greater than 4.15 (using MlogP), and (5) More than three rotatable bonds (NBR) [71, 81]. In this study, the applicability of the rule-of-five was assessed for the hit compounds. **Table 4** presents the results, showing the number of violations for each criterion among the hit compounds compared to standard drugs. Specifically, the **Table 4** includes data on hydrogen-bond donors (HBD), hydrogen-bond acceptors (HBA), the number of rotatable bonds (NBR), molecular weight (MW), and logP values. The analysis indicates that while some of the hit compounds conform to the rule-of-five criteria, others exhibit multiple violations. Compounds with more violations are likely to encounter issues related to absorption and bioavailability. Comparing these results with those of standard drugs provides insight into the relative drug-likeness of the compounds and their potential for effective oral administration. This assessment is critical for guiding the selection of compounds for further development, particularly in optimizing their pharmacokinetic properties to enhance their prospects for clinical success.

The article "Structure-based virtual screening of Trachyspermum ammi metabolites targeting acetylcholinesterase for Alzheimer’s disease treatment" was retracted in 2025. Reasons: unreliable results or conclusions; concerns about the peer review; concerns about the authorship.

**Table 4:** Lipinski’s rule of five parameters for the hit compounds.

Name	HBD	HBA	NBR	LogP	MW	Lipinski Rule	
						Follow	Violation
VIR	1	1	0	3.43	222.3	5	0
PHE	5	7	4	0.61	328.3	5	0
CUR	0	0	4	4.86	202.3	4	1
STE	1	1	0	3.93	248.4	4	1
GAL	1	4	1	1.92	287.3	5	0

HBD = Number of H-bond donors, HBA = Number H-bond acceptors, NBR = Number of rotatable bonds, MW = Molecular weight

### 3.5. ADMET analysis

ADMET screening has become increasingly important in drug development, as it helps reduce the costs and time associated with *in vivo* experiments by evaluating a drug’s absorption, distribution, metabolism, excretion, and toxicity properties early in the process [82]. As shown in **Table 5**, all the identified hit compounds exhibit high human intestinal absorption (HIA) rates, exceeding 90%, with the exception of 2-Methyl-3-glucosyloxy-5-isopropyl phenol, which has a lower absorption rate of 39.61%, indicating poor oral absorption. All the studied compounds were identified as P-glycoprotein inhibitors, which suggests that their absorption will not be hindered by this efflux transporter.

**Table 5:** ADMET properties of hit compounds with comparison to the reference drug.

Name	Absorption		Distribution		Metabolism	Excretion	Toxicity
	HIA	C2P	P-GpI	BBB	CYP2C9	TC	hERG
VIR	92.814	1.483	No	0.632	No	0.817	No
PHE	39.610	-0.219	No	-0.922	No	0.869	No
CUR	93.896	1.555	No	0.599	No	1.511	No
STE	96.204	1.492	No	0.716	Yes	0.955	No
GAL	94.994	1.594	No	-0.081	No	0.991	No

HIA = Human intestinal absorption (%), C2P = CACO-2 permeability (log Papp in 10–6 cm/s), P-GI = P-glyco-protein inhibitor, BBB = Blood-brain barrier (log BB), hERG = human Ether-a-go-go Related Gene, TC = Total Clearance (log ml/min/kg)

In the development of AChE inhibitors, blood-brain barrier (BBB) permeability is a critical factor, as compounds that cannot cross the BBB will not effectively reach neuronal cells in the brain, thus limiting their efficacy as AChE inhibitors [82]. Our study found that three of the identified hits exhibit good BBB permeability compared to the reference drug. However, 2-Methyl-3-glucosyloxy-5-isopropyl phenol was predicted to have poor BBB permeability.

The article "Structure-based virtual screening of Trachyspermum ammi metabolites targeting acetylcholinesterase for Alzheimer’s disease treatment" was retracted in 2025. Reasons: unreliable results or conclusions; concerns about the peer review; concerns about the authorship.

Moreover, none of the compounds were predicted to be hERG inhibitors, suggesting that they are unlikely to pose a risk of cardiotoxicity. hERG inhibition, which can affect potassium channels, is primarily associated with QT syndrome, leading to potential ventricular arrhythmia [83].

### 3.6. DFT based chemical descriptors and analysis

The interaction of a molecule with other species is influenced by its frontier molecular orbitals (FMOs), specifically the highest occupied molecular orbital (HOMO) and the lowest unoccupied molecular orbital (LUMO) (**S3 Fig**). The energy gap between these FMOs plays a crucial role in determining the molecule’s reactivity and stability. A smaller energy gap suggests that the molecule is softer, more polarizable, and typically exhibits higher chemical reactivity but lower kinetic stability. Conversely, a larger energy gap indicates greater molecular stability [84]. In this study, the energy gaps of the identified hit compounds were found to range between 5.98 eV and 8.71 eV, indicating that these compounds are kinetically more stable compared to the reference compound, galantamine, which has a lower energy gap of 4.99 eV (**S4 Fig**).

The MEP map is a valuable tool for predicting sites of hydrogen bonding and understanding biological recognition processes [85, 86]. For all optimized structures of the hit compounds, as well as the control ligand, the reactive sites for electrophilic and nucleophilic attacks were identified using MEP analysis (**S5 Fig**). The positive regions (blue) represent sites suitable for nucleophilic attack, while the negative regions (red) indicate favorable sites for electrophilic interaction, with areas of zero potential appearing in green. The red regions, rich in electrons, are electron-rich, whereas the blue regions are electron-deficient. Hydrogen atoms exhibit the highest positive potential, whereas oxygen atoms show the highest negative potential. Notably, Alpha-Curcumene displayed the lowest electrostatic potential, which corresponds with its lack of hydrogen bonding with the receptor, as observed in the non-bonded interaction analysis of the docking study and the interaction histogram from the MD simulation. These findings offer valuable insights into the stability and reactivity of the hit compounds and their potential interactions with the target receptor, providing a basis for further development as effective inhibitors.

The article "Structure-based virtual screening of Trachyspermum ammi metabolites targeting acetylcholinesterase for Alzheimer’s disease treatment" was retracted in 2025. Reasons: unreliable results or conclusions; concerns about the peer review; concerns about the authorship.

## 4. Conclusion

Computer-assisted virtual screening offers a cost-effective and efficient approach to accelerating the drug development process. In this study, four hit compounds were identified with promising drug-like properties, favorable ADMET and toxicity profiles, and strong binding affinity for the AChE enzyme. MD simulations further confirmed the stability of the receptor-ligand complexes. These findings provide a solid foundation for experimentalists to conduct *in vitro* and *in vivo* studies to validate the AChE inhibitory potential of *Trachyspermum ammi*. If further studies confirm these results, the bioactive compounds from this plant could offer a safe and effective treatment option for Alzheimer’s disease in clinical settings.

## Supporting information

S1 Fig Superimposed structures of cocrystal ligand (Gray), and its re-docked conformer (Green) with an RMSD of 0.077 Å. (DOCX)

S2 Fig Molecular docking scores of 67 compounds. (DOCX)

S3 Fig Frontier molecular orbitals (HOMO and LUMO) of Viridiflorol. (DOCX)

S4 Fig Comparative analysis of chemical reactivity and kinetic stability descriptors. (DOCX)

S5 Fig Electrostatic potential map highlighting deep red regions favorable for electrophilic attack and deep blue regions prone to nucleophilic attack. (DOCX)
